The article "Impact of Femoral Neck Cortical Bone Defect Induced by Core Decompression on Postoperative Stability: A Finite Element Analysis" was published in 2022. Journal: Biomed Res Int.

# Impact of Femoral Neck Cortical Bone Defect Induced by Core Decompression on Postoperative Stability: A Finite Element Analysis

**DOI:** 10.1155/2022/3667891

**Published:** 2022-05-20

**Authors:** Daizhu Yuan, Zhanyu Wu, Siwei Luo, Qiang Zou, Zihao Zou, Chuan Ye

**Affiliations:** ^1^Department of Orthopaedics, The Affiliated Hospital of Guizhou Medical University, Guiyang 550004, China; ^2^Center for Tissue Engineering and Stem Cells, Guizhou Medical University, Guiyang 550004, China; ^3^Sports Medicine, The Affiliated Hospital of Guizhou Medical University, Guiyang 550004, China

## Abstract

**Objective:**

To analyze the impact of femoral neck cortical bone defect induced by core decompression on postoperative biomechanical stability using the finite element method.

**Methods:**

Five finite element models (FEMs) were established, including the standard operating model and four models of cortical bone defects at different portions of the femoral neck (anterior, posterior, superior, and inferior). The maximum stress of the proximal femur was evaluated during normal walking and walking downstairs.

**Results:**

Under both weight-bearing conditions, the maximum stress values of the five models were as follows: femoral neck (inferior) > femoral neck (superior) > femoral neck (posterior) > femoral neck (anterior) > standard operation. Stress concentration occurred in the areas of femoral neck cortical bone defect. Under normal walking, the maximum stress of four bone defect models and its increased percentage comparing the standard operation were as follows: anterior (17.17%), posterior (39.02%), superior (57.48%), and inferior (76.42%). The maximum stress was less than the cortical bone yield strength under normal walking conditions. Under walking downstairs, the maximum stress of four bone defect models and its increased percentage comparing the standard operation under normal walking were as follows: anterior (36.75%), posterior (67.82%), superior (83.31%), and inferior (103.65%). Under walking downstairs conditions, the maximum stress of bone defect models (anterior, posterior, and superior) was less than the yield strength of cortical bone, while the maximum stress of bone defect model (inferior) excessed yield strength value.

**Conclusions:**

The femoral neck cortical bone defect induced by core decompression can carry out normal walking after surgery. To avoid an increased risk of fracture after surgery, walking downstairs should be avoided when the cortical bone defect is inferior to the femoral neck except for the other three positions (anterior, posterior, and superior).

## 1. Introduction

Osteonecrosis of the femoral head (ONFH) is a common clinical disease, and trauma, abuse of immunosuppressants, and long-term excessive alcohol consumption are common pathogenic factors [1, 2]. Inappropriate treatment can lead to the collapse of the femoral head and the destruction of hip joint function. Therefore, hip preservation treatment prior to the collapse of the femoral head (in early ONFH) is very important [3]. Currently, ONFH is mainly treated with core decompression combined with other therapies, such as stem cell transplantation [4], platelet-rich plasma instillation [5], porous tantalum rod implantation [6], and quadratus femoris muscle pedicle bone grafting [7]. These procedures promote the gradual replacement of the dead bone in the necrotic area, tissue repair, and mechanical strength; prevent further collapse of the femoral head; alleviate hip pain; and improve hip joint function.

The article "Impact of Femoral Neck Cortical Bone Defect Induced by Core Decompression on Postoperative Stability: A Finite Element Analysis" was published in 2022. Journal: Biomed Res Int.

For the core decompression of ONFH, a single channel is drilled with a large-diameter hollow drill at an entry point on the outer wall of the tuberosity, inferior to the femoral tuberosity [8]. By drilling through the necrotic tissue sclerosis zone, the high pressure in the femoral head is reduced, and the passage for the growth of new blood vessels in the femoral head is opened up [9]. Core decompression channels through the hardened zone of necrotic tissue to ensure adequate decompression of the necrotic area require consideration of the anatomical characteristics of the proximal femur, including two angle parameters: neck shaft angle and anteversion angle [10]. Core decompression requires conventional positioning of two angle radiography to ensure the safety of the operation, which can be better evaluated by conventional anteroposterior and lateral hip radiographs [11], but it is difficult to achieve in core decompression surgery. The patient was in the supine position during the operation, and anteroposterior radiograph of hip joint can be better displayed as an auxiliary reference for neck shaft angle, but the lateral hip radiographs during the operation are difficult to obtain and display because of anatomic overlap of the healthy proximal femur. Based on this, similar to most literature reports [12, 13], core decompression was assisted by frog position radiography of the hip joint to show proximal femoral anteversion angle during operation. Although frog radiographs of the hip joint can better assist the positioning of anteversion angle, we found in clinical practice that well-positioned frog radiographs of core decompression showed injury to the cortical bone of the femoral neck (Figure 1), and it has been verified through the model that core decompression with frog position assisted positioning anteversion angle may injury different positions of femoral neck cortical bone (Figure 2). There is a narrow area of physiological diameter in the proximal femoral neck [14]; when the cortical bone was damaged by core decompression, the cortical bone structure in the femoral neck narrow area was the first injured. Compared to cancellous bone, cortical bone has a denser texture and greater resistance to compression and distortion and is distributed on the surface of the bone, which is important for the mechanical support of the entire body [15]. Core decompression damages the cortical bone at the narrow region of the femoral neck, causing changes in the original mechanical structure and local concentration of stress, which can cause local bone defects and reduced mechanical strength. The bone defect can result in mechanical instability and may reduce the load that bone can bear compared to normal bone, which may even increase the risk of local fractures. Studies have shown that local bone defects of the acetabulum can affect local biomechanical properties, and bone defects should be repaired during joint replacement to ensure initial postoperative stability [16]. Partial bone loss of the glenoid cavity leads to bone defect and mechanical stability decline, which requires local bone fixation to enhance the stability of the shoulder joint [17]. The previous study showed that nonstandard core decompression operation may even lead to an increased risk of proximal femoral fractures [18]. Whether there are differences in mechanical properties of bone defects in different positions, existing literature has reported the mechanical properties of bone defects caused by bone tumors at different parts of the proximal femur, indicating that the stiffness value of the medial defect group is significantly lower than that of the intact femur, and the axial failure strength is lower than that of the anterior and posterior position groups [19]. Zhang et al. established different bone defect models of proximal femur by finite element method and analyzed the stress changes of bone defect in proximal femur region, intertrochanteric region, and femoral neck by simulating the loading of walking load. The results showed that the location and size of bone defect would affect the local biomechanical strength and the degree of fracture risk at different locations [20]. Some scholars have analyzed whether the local bone defect area will lead to fracture after the treatment of femoral head necrosis with greater trochanter bone flap transfer. The results showed that there was local stress concentration in the bone defect area, but the risk of local fracture did not increase [21]. The bone tunnel can be understood as a local bone defect on the bone surface. Some studies have analyzed the safety diameter parameters of core decompression at different positions proximal to the femur, and the results show that the safety parameter range of drilling location under the lesser trochanter is the smallest, and the risk of fracture is the highest [22]. Bonano et al. analyzed the influence of local bone defect of the femoral neck after femoroacetabular impingement on postoperative biomechanics through finite element analysis, indicating that the depth of local bone defect is related to the risk of postoperative fracture [23], and there have been studies that have shown the risk of fracture after surgery [24]. To prevent the risk of recurring fractures, clinicians tell patients to avoid early weight-bearing activities based on subjective experience, but the relationship between early weight-bearing activities and mechanical instability is not clear [25]. This leads to the recommendation that patients with damage to the femoral neck cortex or local bone defects caused by core decompression avoid early weight-bearing activities, and patients do not receive appropriate guidance regarding the appropriate duration and intensity of weight-bearing activities with crutches. There are still few studies on whether there are differences in mechanical properties of cortical bone injury or even bone defect at different locations of the femoral neck.

The article "Impact of Femoral Neck Cortical Bone Defect Induced by Core Decompression on Postoperative Stability: A Finite Element Analysis" was published in 2022. Journal: Biomed Res Int.

In this study, we analyzed the biomechanical impact of bone defects at different portions of the femoral neck cortical bone caused by core decompression and determined whether the daily activities of normal walking and walking downstairs after surgery affect the mechanical stability of the proximal femur, which identify a “safe zone” and guide the clinical application.

## 2. Materials and Methods

### 2.1. Construction of Three-Dimensional (3D) Femur Model and Early ONFH

A 3D model of the Sawbones® left fourth-generation composite femur (Model 3406; Sawbones, Vashon, WA) was used for the geometric model of the femur, including femoral cortical and cancellous bones (Figure 3(a)). Then, we constructed the early ONFH using the SolidWorks 2018 software (Dassault, France). The necrosis area was determined based on the angles in the midcoronal and midsagittal images of the femur. Both angles were set at 100° corresponding to the extent of early ONFH [26] (Figure 3(b)).

### 2.2. Construction of Different Core Decompression Models

Five types of FEMs were constructed using the SolidWorks 2018 software. Eight-millimeter-diameter hollow core drill decompression, a conventional clinical application [27], served as the standard operating model (Figure 4(a)). The remaining four femoral neck defect models were based on the same core drill diameter and drilling angle used in the standard operating model. Models of cortical bone defects at the anterior, posterior, superior, and inferior femoral neck were established at the narrowest position of the femoral neck (Figures 4(b), 4(c), 4(e), and 4(f)). In order to ensure the consistency of the four femoral neck injury models, all cortical bone defects were set to the elliptical shape with a diameter of 4 × 8 mm (parameters simulated hollow core drill exposed half and resulted in bone defect) (Figure 4(d)).

The article "Impact of Femoral Neck Cortical Bone Defect Induced by Core Decompression on Postoperative Stability: A Finite Element Analysis" was published in 2022. Journal: Biomed Res Int.

### 2.3. Finite Element Biomechanical Analysis

The solid models were discretized into ten-node tetrahedral elements (solid 187) using the ANSYS Workbench 2021 software (ANSYS, American). We performed a sensitivity analysis to determine the appropriate element size for our model [28, 29]. The standard operating model was used to construct FEMs comprising five different element sizes (1.5, 2, 3, 4, and 5 mm). Then, the maximum equivalent stress in the femoral neck area of the models with five different element sizes was compared. The percentage change in the normal walking load between the 1.5 mm model and the 2 mm model was 0.4%. The percentage change between the 2 and 3 mm models, 2 and 4 mm models, and the 2 and 5 mm models were 4.2%, 8.4%, and 12.5%, respectively. Even the finest mesh (1.5 mm) did not result in a significant percentage difference. Therefore, the 2 mm mesh was used for the FEMs. There were approximately 410,000 nodes (from 413,967 to 420,753) and 280,000 elements (from 281,095 to 281176) in each model (Table 1). All materials were assumed to be homogeneous, isotropic, and with linear elastic behavior [30, 31] (Table 2). The type of mechanical contact between the cortical and cancellous bone was bonded [32]. Two types of mechanical loads—normal walking and walking downstairs—were assigned to the femoral head according to a previous study [33] (Table 3). The load was applied in a distributed manner on the femoral contact area in order to simulate the actual behavior of the joint. The contact area was set as the contact surface of the acetabular cartilage (weight-bearing area: the angle between the front and back directions of the femoral head surface and the center of the femoral head was 80°, and the angle between the inside and outside directions of the surface of the femoral head and the center of femoral head was 40° [34]). The distal end of the femur was constrained.  Figure 5 shows models of the femur which detail the area where the load was applied and the area in which the constraint was applied.

The article "Impact of Femoral Neck Cortical Bone Defect Induced by Core Decompression on Postoperative Stability: A Finite Element Analysis" was published in 2022. Journal: Biomed Res Int.

### 2.4. Evaluation Indices

The stress distributions and maximum stress of the proximal femur were evaluated during normal walking and walking downstairs.

## 3. Results and Discussion

### 3.1. Stress Distribution of the Femoral Neck Cortical Bone

As shown in Figure 6, the stress in the femoral neck region was uniformly distributed in the standard operating model, with the maximum stress region located inferior to the femoral neck. Under normal circumstances, the load transmitted from the femoral head to the femoral neck is not in a straight line due to the femoral neck shaft angle and anterior angle, resulting in tension, pressure, and shear force at the femoral neck, which is mainly concentrated at the lower part of the femoral head-neck joint [35]. This was similar to those of our study, and the same mechanism was applicable to our study, showing that the standard operating model does not alter the stress distribution in the femoral neck region. However, as can be seen from Figures 7 and 8, in the other four cortical bone defect models, the stress concentration was distributed around the cortical bone defect of the femoral neck, and all four models had more significant stress concentration than the standard operating model. Among cortical bone defect models, the stress concentration of the inferior femoral neck defect model was most significant, followed by femoral neck (superior), femoral neck (posterior), and femoral neck (anterior). Human bone is an elastic material, and plastic deformation occurs when it is subjected to external stress [36], which can change the distribution of stress. In this study, core decompression damaged the cortical bone in the narrow region of the femoral neck, causing changes in the original mechanical structure and stress distribution change.

### 3.2. Stress Distribution under the Condition of Normal Walking

Under the normal walking condition, the maximum equivalent stress of the standard operation model was 51.18 MPa, and those of the cortical bone defect models were 59.97 MPa for the femoral neck (anterior) model, 71.15 MPa for the femoral neck (posterior) model, 80.60 MPa for the femoral neck (superior) model, and 90.29 MPa for the femoral neck (inferior) model. The maximum stress of four bone defect models and its increased percentage comparing the standard operation were as follows: anterior (17.17%), posterior (39.02%), superior (57.48%), and inferior (76.42%) (Table 4). Results showed that femoral neck (inferior) > femoral neck (superior) > femoral neck (posterior) > femoral neck (anterior). Previous studies have also demonstrated that the stress transmitted downward through the femoral head is mainly distributed in the lower part of the femoral neck (the pressure side) and is also the main fracture site as the load increases [35]. As shown in Figure 7, there was a bone defect on the pressure side of the cortical bone defect model at the lower part of the femoral neck. The stress passing through this region could not be well dispersed and would be concentrated near the bone defect area, resulting in an increase of local stress, which was significantly larger than the other three femoral neck bone defect models. As shown in Figure 7(e), the maximum equivalent stress in the femoral neck region was less than the yield strength value of the cortical bone (104 MPa) [37]. The results showed that under the normal walking load, daily walking activities could be carried out without increasing the risk of postoperative fracture, even though local bone defects in different positions of the femoral neck cortical bone after core decompression. The bone tunnel entry after core decompression was similar to the bone defect. Yuan et al. studied the biomechanical effects of different drilling parameters of bone tunnels under walking load and obtained safe drilling parameters to avoid local fractures [22]. The bone defect caused by a single large diameter bone tunnel can reduce local biomechanical strength; relevant studies have only analyzed stress under walking and stair-climbing conditions after small-diameter multiporous core decompression and found that walking and stair-climbing can be carried out after core decompression [38].

The article "Impact of Femoral Neck Cortical Bone Defect Induced by Core Decompression on Postoperative Stability: A Finite Element Analysis" was published in 2022. Journal: Biomed Res Int.

As can be seen from Table 4, for the maximum stress of the entry area on the outer wall of the femoral trochanter, the standard operating model was lower than that of the femoral neck (anterior) and femoral neck (inferior) defect models, while higher than that of the femoral neck (posterior) and the femoral neck (superior) defect models. These results indicated that drilling position close to the anterior trochanter and the inferior lesser trochanter leads to stress concentration at the entry area, while stress can be distributed evenly and stress shielding can be prevented when the drilling position is close to the posterior trochanter and the superior lesser trochanter (Figure 9). During core compression, a lateral trochanteric approach is made by drilling one single channel with a large-diameter bone tunnel [8]. The lateral wall of the femur is cortical bone, which is denser than cancellous bone, with stronger resistance to compression and distortion, and thus is essential for the mechanical support of the entire body [39]. The core decompression damaged the cortical bone on the lateral wall, causing damage to the original mechanical structure and a decline in its mechanical strength. Studies have shown that the integrity of the lateral wall of the trochanter is important for maintaining the biomechanical stability of the proximal femur [40]. Drilling bone tunnel at the different locations on the lateral wall results in changes in the mechanical strength of local bones and even increases the risk of fractures. It was reported that during the core decompression combined with tantalum rod implantation for early stage osteonecrosis of the femoral head, subtrochanteric fracture occurred after surgery due to drilling location below the lesser trochanter [41]. Cannulated screws were inserted into different locations on the lateral wall of the femoral trochanter in an inverted triangle arrangement for finite element analysis; the results showed that the upper location induced the lowest stress level while the lower location induced the highest stress level, and stress shielding occurred [42]. Femoral subtrochanteric appears stress concentration phenomenon related to the anatomy and biomechanical properties: The stress concentration below the trochanter of the femur is related to its anatomical region and biomechanical properties: this region is the focus of many muscles, such as the adductor, gluteus muscles, iliopsoas, and external rotators. In the subtrochanteric region of the femur, these muscle groups form an area of high mechanical stress by increasing the pressure of the medial cortex and the tension of the lateral bone [43]. The findings are similar to those of our study, and the same mechanism is applicable to our study.

The article "Impact of Femoral Neck Cortical Bone Defect Induced by Core Decompression on Postoperative Stability: A Finite Element Analysis" was published in 2022. Journal: Biomed Res Int.

### 3.3. Stress Distribution under the Condition of Walking Downstairs

Under the walking downstairs condition, the stress concentration in the cortical bone of the femoral neck was similar to that under the normal walking condition. However, the maximum equivalent stress for each model increased to varying degrees: the values were 59.75 MPa for the standard operating model, 69.99 MPa for the femoral neck (anterior), 85.89 MPa for the femoral neck (posterior), 93.82 MPa for the femoral neck (superior), and 104.23 MPa for the femoral neck (inferior). The maximum stress of four bone defect models and its increased percentage comparing the standard operation under normal walking were as follows: anterior (36.75%), posterior (67.82%), superior (83.31%), and inferior (103.65%) (Table 4).

Under the walking downstairs condition, the maximum stress of bone defect models (anterior, posterior, and superior) was less than the yield strength of cortical bone, while the bone defect model (inferior) excessed yield strength value. The results showed that walking downstairs should be avoided to prevent the risk of postoperative fracture when the cortical bone defect is inferior to the femoral neck except for the other three positions (anterior, posterior, and superior). Studies have analyzed the stress distribution in the tunnel entrance area and the risk of fracture after core decompression using the same load as ours [18]. However, the position of analysis differs from that of this study. As can be seen in Figure 8, under the walking downstairs load, research suggested the presence of obvious stress concentration in the defect area of the femoral neck cortical bone. Bone tissue produces stress under the action of external force. When stress concentration occurs in a certain area of bone, local stress or strain exceeds the ultimate stress or ultimate strength of this area, bone tissue material is damaged, and fracture occurs [44]. Therefore, the pattern of stress and the structural characteristics of bone determine the occurrence and prognosis of fracture. As can be seen from Figure 8(e), the maximum stress of the bone defect model (inferior) excessed cortical bone yield strength, showing that the bone defect at this location shows significant stress concentration and increases the risk of postoperative fracture. Studies have shown that stress concentration is often the starting point for the destruction that reduces strength and load-bearing capacity [45]. One of the main complications of bone defect is a fracture; the larger the bone defect, the greater the risk of fracture, including the size and location of the defect [46].

The article "Impact of Femoral Neck Cortical Bone Defect Induced by Core Decompression on Postoperative Stability: A Finite Element Analysis" was published in 2022. Journal: Biomed Res Int.

The maximum stress values at the entry area of the different drilling locations of the five models were as follows: femoral neck (anterior) (64.62 MPa) > femoral neck (inferior) (38.54 MPa) > standard operation (32.70 MPa) > femoral neck (superior) (27.0 MPa) > femoral neck (posterior) (20.28 MPa) (Table 4). As can be seen from Figure 9, the stress distribution in the tunnel entrance area is similar to that under normal walking conditions. Under the two daily activities of normal walking and walking downstairs, the stress level at the entry area in the femoral neck (anterior) defect model was significantly higher than that in the femoral neck (posterior) defect model. This may be related to the anatomical features of the femoral trochanter. The anterior femoral trochanter is relatively flat, and the posterior femoral trochanter is connected to the lesser trochanter, which protrudes backward [47]. As shown in Figures 8(a) and 9(a) of this study, core decompression damaged the cortical bone of the anterior femoral neck and led to damaging cortical bone structures of the femoral anterior trochanter due to the lack of a good transitional structure between the flat anterior trochanter and the narrow area of the femoral neck. On the other hand, in the femoral neck (posterior) defect model, the excellent structural transition between the posteriorly protruding lesser trochanter and the narrow area of the femoral neck ensured that the cortical bone structure of the posterior trochanter was not affected by the damage of the cortical bone at the narrow area of the posterior femoral neck after core decompression. As a result, as shown in Figures 8(b) and 9(b), the stress at the entry area was low, and stress shielding was prevented.

The article "Impact of Femoral Neck Cortical Bone Defect Induced by Core Decompression on Postoperative Stability: A Finite Element Analysis" was published in 2022. Journal: Biomed Res Int.

A limitation of this study was that the material properties are assumed to be isotropic, linearly elastic, and homogeneous. We ignored the soft tissue surrounding the proximal femur. This study only considered the commonly used 8 mm diameter hollow core drill and did not analyze other types. Moreover, the bone defect was only studied in half cases of exposure, not in all cases.

## 4. Conclusions

The femoral neck cortical bone defect induced by core decompression can carry out normal walking after surgery. To avoid an increased risk of fracture after surgery, walking downstairs should be avoided when the cortical bone defect is inferior to the femoral neck except for the other three positions (anterior, posterior, and superior).

## Figures and Tables

**Figure 1:** Clinical findings. (a) Conventional anteroposterior (a1) and lateral hip radiographs (a2) showing the neck shaft angle and anteversion angle. (b) Positioning of anteroposterior (b1) and frog position radiograph (b2) during core decompression. (c) Radiographs of injuring the cortical bone during surgery. (c1) Anteroposterior radiograph shows the good position of core decompression. (c2) Frog position radiograph shows the positioning to be slightly forward and does not exceed the bony margin of the femoral neck, while the cortical bone has been injured (red oval). (c3) Bone structure showing damaged femoral neck cortical bone (yellow arrow).

**Figure 2:** Frog position radiograph assisted positioning anteversion angle injury different positions of femoral neck cortical bone during core decompression (i: anteroposterior radiograph showing cortical bone injury-blue oval; ii: frog position radiograph showing no cortical bone injury-blue oval): (a) radiographic positioning of conventional core decompression; (b) radiographic positioning of anterior cortical bone injury; (c) radiographic positioning of posterior cortical bone injury; (d) radiographic positioning of superior cortical bone injury; (e) radiographic positioning of inferior cortical bone injury.

**Figure 3:** Construction of 3D models: (a) femoral cortical and cancellous bone; (b) necrotic area of early ONFH.

The article "Impact of Femoral Neck Cortical Bone Defect Induced by Core Decompression on Postoperative Stability: A Finite Element Analysis" was published in 2022. Journal: Biomed Res Int.

**Figure 4:** Construction of different core decompression models (yellow: cortical bone, blue: cancellous bone, red: necrotic area, green: bone defect): (a) standard operating model without cortical bone injury; (b) femoral neck (anterior) defect with cortical bone injury; (c) femoral neck (posterior) defect with cortical bone injury; (d) size of the bone defect; (e) femoral neck (superior) defect with cortical bone injury; (f) femoral neck (inferior) defect with cortical bone injury.

**Figure 5:** Meshing and boundary conditions: (a) meshed model of proximal femur; (b) contact region setting; (c) contact loading (normal walking and walking downstairs).

**Figure 6:** Stress distribution of the standard operating model: (a, b) femoral neck cortical bone under normal walking and walking downstairs; (c, d) entry area of bone tunnel under normal walking and walking downstairs.

**Figure 7:** Stress distribution of the cortical bone defects under normal walking: (a) femoral neck (anterior) defect; (b) femoral neck (posterior) defect; (c) femoral neck (superior) defect; (d) femoral neck (inferior) defect; (e) maximum stress versus yield strength.

**Figure 8:** Stress distribution of the cortical bone defects under walking downstairs: (a) femoral neck (anterior) defect; (b) femoral neck (posterior) defect; (c) femoral neck (superior) defect; (d) femoral neck (inferior) defect; (e) maximum stress versus yield strength.

**Figure 9:** Stress distribution at the entry area: (a) femoral neck (anterior) defect; (b) femoral neck (posterior) defect; (c) femoral neck (superior) defect; (d) femoral neck (inferior) defect under normal walking and walking downstairs (e–h); (i) maximum stress at the entry area under normal walking and walking downstairs.

**Table 1:** Notes and elements of models in this study.

	Standard	Anterior	Posterior	Superior	Inferior
Notes	419679	419750	420753	413967	420425
Elements	280364	280684	281176	281095	280772

**Table 2:** Material properties of all modes in this study.

Materials	Young's modulus (MPa)	Poisson's ratio
Cortical bone	15100	0.3
Cancellous bone	445	0.22
Early ONFH	332.9	0.3
Articular cartilage	150	0.2

**Table 3:** Force components and resulting forces for the load cases of normal walking and walking downstairs.

	Components and resultant forces (N)			
Load cases	*F*_*x*_	*F*_*y*_	*F*_*z*_	∣*F*∣
Normal walking	−405.8	247.5	2017.0	2072.3
Walking downstairs	−533.2	344.0	2369.3	2452.8

**Table 4:** The maximum equivalent stress of different models and increased/decreased percentage comparing the standard operation under normal walking.

Models	The area of femoral neck cortical bone defect (MPa)	The entry area of drilling location (MPa)
Normal walking		
Standard operation	51.18	29.55
Femoral neck (anterior)	59.97 (17.17%)	55.44 (87.61%)
Femoral neck (posterior)	71.15 (39.02%)	19.57 (-33.77%)
Femoral neck (superior)	80.60 (57.48%)	24.44 (-17.29%)
Femoral neck (inferior)	90.29 (76.42%)	35.06 (18.65%)
Walking downstairs		
Standard operation	59.75 (16.74%)	32.70 (10.66%)
Femoral neck (anterior)	69.99 (36.75%)	64.62 (118.68%)
Femoral neck (posterior)	85.89 (67.82%)	20.28 (-31.37%)
Femoral neck (superior)	93.82 (83.31%)	27.00 (-8.63%)
Femoral neck (inferior)	104.23 (103.65%)	38.54 (30.42%)

The article "Impact of Femoral Neck Cortical Bone Defect Induced by Core Decompression on Postoperative Stability: A Finite Element Analysis" was published in 2022. Journal: Biomed Res Int.

## Data Availability

All data analyzed during this study are included in this article.
